# Cervical Cytology of Samples with *Ureaplasma urealyticum*, *Ureaplasma parvum*, *Chlamydia trachomatis*, *Trichomonas vaginalis*, *Mycoplasma hominis*, and *Neisseria gonorrhoeae* Detected by Multiplex PCR

**DOI:** 10.1155/2020/7045217

**Published:** 2020-07-07

**Authors:** Fabiana Pirani Carneiro, Andersen Charles Darós, Adriana Cysneiro Milhomem Darós, Tércia Maria Mendes Lousa de Castro, Marcos de Vasconcelos Carneiro, Cecília Ramos Fidelis, Mariane Vieira Vilioni, Michelle Egídio da Costa Matsunaga, Jéssica Meneses Othon Sidou, Mariana Anaue Lozi Dias Chaves, Lívia Custódio Pereira, Ceres Nunes de Resende, Agenor de Castro Moreira dos Santos, Vânia Moraes Ferreira, Andrea Barretto Motoyama

**Affiliations:** ^1^Pathology Department of Brasília University, Brasília, Federal District, Brazil; ^2^Catholic University of Brasilia, Brasília, Federal District, Brazil; ^3^Gynecological Unit, University Hospital of Brasilia, Brasília, Federal District, Brazil; ^4^Molecular Biology Laboratory-LACEN DF, Brazil

## Abstract

**Introduction:**

Despite increasing application of molecular diagnostic methods for the detection of sexually transmitted infections, the cytological findings in pap smears of patients with pathogens that can be identified only by PCR are not yet well described. The aim of this study was to describe the most common cytological features in cervical pap smears of patients with *Chlamydia trachomatis*, *Neisseria gonorrhoeae*, *Mycoplasma genitalium*, *Trichomonas vaginalis*, *Mycoplasma hominis*, *Ureaplasma urealyticum*, and *Ureaplasma parvum* detected by multiplex PCR.

**Methods:**

Cervical samples for conventional and liquid-based cytology and for multiplex PCR were collected from women ranging from 23 to 54 years old, who underwent routine screening at a gynecological Unit.

**Results:**

Multiplex PCR was positive in 36.2% of the samples: *Ureaplasma parvum* 14.9%, *Chlamydia trachomatis* 10.6%, *Trichomonas vaginalis* 10.6%, *Mycoplasma hominis* 8.5%, *Ureaplasma urealyticum* 4.2%, *Neisseria gonorrhoeae* 2.1%, and *Mycoplasma genitalium* (0). Multiple pathogens were observed in 12.8% of samples. Microscopic cervicitis (≥10 polymorphonuclear leukocytes/epithelial cell) and normal (predominantly lactobacillary) microbiota were the most frequent findings in the samples in which the pathogens were detected alone or in multiple infections, except for samples with *Trichomonas vaginalis* in which the coccobacillary microbiota was the most common. In samples with microscopic cervicitis and normal microbiota, those with at least one pathogen identified by multiplex PCR were significantly more frequent than those with no pathogen, 66.6% versus 33.3%.

**Conclusion:**

Failure to identify an inflammatory agent in pap smear with intense neutrophil exudate may suggest the presence of *Ureaplasma parvum*, *Ureaplasma urealyticum*, *Chlamydia trachomatis*, or *Trichomonas vaginalis*. A remark on the intensity of inflammation should be made in the reports of cervical pap smears so that this cytological finding can be correlated with clinical and PCR results.

## 1. Introduction

Cervicitis is a common, often symptomatic, and clinically relevant disease [1]. Complications of cervicitis include endometritis, pelvic inflammatory disease, and adverse outcomes in pregnancy and to the newborn [1]. Cervicitis is also associated with enhanced risk for HIV (Human Immunodeficiency Virus) and HPV (Human Papillomavirus) transmission and for cervical cancer development [1]. Cervicitis definitions with best clinical utility and pathogen prediction were those based on clinical assessments (mucopurulent cervical discharge) and microscopic findings: >30 pmnl/hpf (polymorphonuclear leukocytes per high-powered field) on Gram stain [2].

*Chlamydia trachomatis* and *Neisseria gonorrhoeae* have been considered the major causes of cervicitis; however, these pathogens account for less than 50% of cervicitis cases [3]. In the remaining cases, the disease is termed nonchlamydial and nongonococcal cervicitis or nonspecific cervicitis, and the organisms involved may include Mycoplasma species, Ureaplasma species, herpes simplex virus, cytomegalovirus, and *Trichomonas vaginalis* [4, 5]. With the implementation of nucleic acid amplification tests (NAATs), the detection of these pathogens has been performed with elevated specificity and sensitivity, and by multiplex PCR, they can be detected simultaneously [6].

The Papanicolaou (pap) smear test is a simple, quick, low-cost, and painless procedure used as a screening test for the prevention of cervix cancer. Although according to the current Bethesda system it is not mandatory to report the presence of microorganisms or other nonneoplastic findings, usually, when reporting the results of cervical pap smear tests, a remark is made on their presence on cytological criteria [7]. The main advantage of the use of the pap smear as a presumptive diagnostic method is the fact that it is a routine test widely used to which a very large number of women are still periodically submitted. In developing countries, for diagnosis of cervicovaginal infections, clinical examination and pap smear are, often, the only available exams.

Despite increasing application of molecular diagnostic methods for the detection of sexually transmitted infections, the cytological findings in pap smears of patients with pathogens that can be identified only by PCR or culture are not yet well described in the literature. The aim of this study is to describe the most common cytological features in cervical pap smears of patients with *Chlamydia trachomati*s, *Neisseria gonorrhoeae*, *Mycoplasma genitalium*, *Trichomonas vaginalis*, *Mycoplasma hominis*, *Ureaplasma urealyticum*, and *Ureaplasma parvum* detected by multiplex PCR.

## 2. Materials and Methods

### 2.1. Study Design and Eligibility

The study population consisted of women, ranging from 23 to 54 years old, who underwent routine screening in 2017–2018 at a gynecological clinic. Eligible criteria included (i) age ≥ 18 years, (ii) no use of antibiotic therapy 12 months prior to sample collection, and (iii) no topical medications in the previous month.

### 2.2. Cytology

For conventional preparations (CP), samples were collected from the ectocervix and endocervix with Ayre's spatula and cytobrush, respectively. The smears were immediately fixed in 99% ethanol and stained by the Papanicolaou method.

For liquid-based preparations (LBP), samples were collected from the endocervix with a cytobrush that was rinsed in ThinPrep® PreservCyt® Solution. The solution was centrifuged, and only 1 mL of the solution was left with the pellet. About 200 *μ*L of concentrated sample were cytocentrifuged for each slide. The slides were stained by the Papanicolaou method. The smears were analyzed by one pathologist who was blinded to the PCR results.

The criterion for microscopic cervicitis was established by using five samples from patients with mucopurulent discharge, clinically defined by an experienced gynecologist. In liquid-based preparations, the number of polymorphonuclear leukocytes (pmnl) was counted in at least 10 representative high-powered field (hpf) (400x), and the lower mean was about 10 pmnl/epithelial cell. Thus, it was considered microscopic cervicitis when the (mean) number of pmnl/epithelial cell was higher than or equal to 10 (≥10 pmnl/epithelial cell), in at least 10 hpf (Figure 1).

Lactobacilli were characterized by the presence of elongated bacillary structures. Coccobacilli, characterized by small bacilli and cocci organisms, were found both isolated and as microcolonies. Individual squamous cells with a layer of coccobacilli along the margins of the cell membranes (supracytoplasmic bacilli) were considered “clue cells.” Samples with *Candida sp*, actinomyces, and cellular changes consistent with the herpes simplex virus and with the cytomegalovirus were excluded from the study. Samples with coccobacillary microbiota were excluded from the comparison analysis of the presence of cervicitis in samples with and without pathogen.

The cytological abnormalities were classified according to the current Bethesda system into the following categories: (i) negative, (ii) atypical squamous cells of undetermined significance (ASC-US), (iii) atypical glandular cells (AGC), (iv) atypical squamous cells-cannot exclude high-grade intraepithelial lesion (ASC-H), (v) low-grade squamous intraepithelial lesion (LSIL), (vi) high-grade squamous intraepithelial lesion (HSIL), (vii) squamous cell carcinoma, (viii) adenocarcinoma *in situ*, and (ix) invasive adenocarcinoma [7].

### 2.3. Pathogen DNA Extraction

Pathogen DNA extraction was performed from cervical swabs using the PureLink Microbiome DNA Isolation kit (Thermo Fisher), according to the manufacturer's instructions. In brief, the preserved brushes were heated to 65°C/10 min in a solution containing lysis buffer, beads, and 2 *μ*L of the internal control for qPCR (provided by the qPCR detection kit manufacturer). Immediately after incubation, the samples were subjected to vigorous vortexing for 10 min. After centrifugation, the supernatant was passed through a column and washed several times with the buffers provided, and the DNA was eluted in 50 *μ*L of elution buffer.

### 2.4. Multiplex qPCR

A multiplex PCR was performed to detect the presence of *Chlamydia trachomatis* (CT), *Neisseria gonorrhoeae* (GC), *Mycoplasma genitalium* (MG), *Trichomonas vaginalis* (Tvag), *Mycoplasma hominis* (Mhom), *Ureaplasma urealyticum* (Uurea), and *Ureaplasma parvum* (Uparv), using the XGen Uretrite Plus kit (Mobius Life, Brazil), which is qualitative and not quantitative. The reaction was performed according to the manufacturer's instruction. From each sample, 10 *μ*L was added to a reaction tube containing primers, probes, and the qPCR system for simultaneous detection of either *Neisseria gonorrhoeae*, *Mycoplasma genitalium*, *Chlamydia trachomatis*, and *Trichomonas vaginalis*, simultaneously, or *Ureaplasma urealyticum*, *Ureaplasma parvum*, *Mycoplasma hominis*, and an internal control (a mouse cytomegalovirus sequence), also simultaneously. Thus, each sample was used in two detection tubes, each with probes labelled with the fluorophores FAM, VIC, ROX, and CY5. For the qPCR reaction, positive and negative controls provided in the kit were used. The reaction protocol was 42°C/15 min, 94°C/3 min, and 40 cycles of 94°C/8 sec and 64°C/34 sec, which was performed in a LightCycler 480 Instrument II (Roche). The specificity of the test for each pathogen is 100%, and the sensitivity varies from 10^2^ copies per mL to 10^4^ copies per mL, depending on the microorganism: 10^3^, 10^3^, 10^4^, 10^2^, 10^3^,10^3^, and 10^2^ copies/mL, respectively, for *Chlamydia trachomatis* (CT), *Neisseria gonorrhoeae* (GC), *Mycoplasma genitalium* (MG), *Trichomonas vaginalis* (Tvag), *Mycoplasma hominis* (Mhom), *Ureaplasma urealyticum* (Uurea), and *Ureaplasma parvum* (Uparv). The mean (SD) (min–max) of Cq values of the positive controls was 30.7 (0.95) (29.17-31.69), 30.6 (0.38) (30.25-31.25), 29.8 (0.38) (29.41-30.44), 30.4 (0.54) (29.6-30.83), 29.7 (0.43) (28.98-30.04), 30.3 (1.06) (28.59-31.36), and 31.3 (2.10) (28.04-33.69) for *Chlamydia trachomatis* (CT), *Neisseria gonorrhoeae* (GC), *Mycoplasma genitalium* (MG), *Trichomonas vaginalis* (Tvag), *Mycoplasma hominis* (Mhom), *Ureaplasma urealyticum* (Uurea), and *Ureaplasma parvum* (Uparv), respectively. These mean Cq values for positive controls are below the recommended cut-off Cq of 33 cycles, above which the assay should be deemed invalid.

### 2.5. Statistical Analysis

Statistical analysis was performed with GraphPad Prism 4 (GraphPad Software, San Diego, CA). The Fisher test was used, and statistical significance was assigned to p < 0.05.

## 3. Results

### 3.1. Pathogens Identified by Multiplex PCR

Multiplex PCR was positive in 36.2% (17/47) of the samples as shown in Table 1. Six of the seven different species were identified: *Ureaplasma parvum* 14.9% (7/47), *Chlamydia trachomatis* 10.6% (5/47), *Trichomonas vaginalis* 10.6% (5/47), *Mycoplasma hominis* 8.5% (4/47), *Ureaplasma urealyticum* 4.2% (2/47), and *Neisseria gonorrhoeae* 2.1% (1/47). *Mycoplasma genitalium* was not detected. Multiple pathogens were observed in 12.8% (6/47) of the samples.

### 3.2. Cytological Findings in Cervical Pap Smear

#### 3.2.1. Ureaplasma

*Ureaplasma parvum* was the sole detected pathogen by multiplex PCR in four samples (samples 1 to 4) (Table 1). All samples showed microscopic cervicitis (≥10 pmnl/epithelial cell). Numerous polymorphonuclear leukocytes, isolated or in aggregates (“polyballs”), were observed (Figures 2(a) and 2(b)). The microbiota was normal (predominantly lactobacillary) in 3 samples and with supracytoplasmic bacilli (clue cells) in one sample (Table 1, Figures 2(a) and 2(b)). Reactive-reparative cellular changes were also present.

*Ureaplasma urealyticum* was the sole detected pathogen by multiplex PCR in samples 5 and 6 (Table 1). Microscopic cervicitis with numerous polymorphonuclear leukocytes, isolated or in aggregates (“polyballs”), was observed (Figures 2(c) and 2(d)).The microbiota was normal (predominantly lactobacillary) in one sample and with supracytoplasmic bacilli (clue cells) in the other (Table 1, Figures 2(c) and 2(d)). Reactive-reparative cellular changes were also present.

#### 3.2.2. *Chlamydia trachomatis*

*Chlamydia trachomatis* was the sole detected pathogen by multiplex PCR in three samples (samples 7 to 9) (Table 1). All samples showed microscopic cervicitis with numerous polymorphonuclear leukocytes, isolated or in aggregates (“polyballs”) (Figures 2(e) and 2(f)). The microbiota was normal (predominantly lactobacillary) in two samples and predominantly coccobacillary in one (Table 1, Figures 2(e) and 2(f)). Reactive-reparative cellular changes were also present.

#### 3.2.3. *Trichomonas vaginalis*

*Trichomonas vaginalis* was the sole detected pathogen by multiplex PCR in samples 10 and 11 (Table 1). These two samples showed microscopic cervicitis with numerous polymorphonuclear leukocytes, isolated or in aggregates (“polyballs”). The microbiota was predominantly coccobacillary in one sample and normal (predominantly lactobacillary) in another (Table 1, Figures 2(g) and 2(h)). Only in sample 10 were pear-shaped organisms with an eccentrically located nucleus and eosinophilic cytoplasmic granules, consistent with *Trichomonas vaginalis*, present (Figure 2(h)). In sample 10, HSIL was observed (Figure 2(h)). Reactive-reparative cellular changes were also present.

#### 3.2.4. Multiple Pathogens

*Mycoplasma hominis* was detected with *Trichomonas vaginalis* (samples 13 and 14) with *Ureaplasma parvum* (sample 15) and with both these pathogens (sample 12) (Table 1). In samples 12, 13, and 14, the cytological findings were similar to those of the samples in which *Trichomonas vaginalis* was the sole pathogen detected: microscopic cervicitis with numerous polymorphonuclear leukocytes, isolated or in aggregates (“polyballs”); in samples 12 and 14, the microbiota was predominantly coccobacillary (Figures 3(a) and 3(b)); and in sample 13, it was normal (predominantly lactobacillary) (Table 1). Only in sample 14 were pear-shaped organisms with an eccentrically located nucleus and eosinophilic cytoplasmic granules, consistent with *Trichomonas vaginalis*, present (Figure 3(a)). In sample 14, HSIL was observed (Figure 3(a)). In sample 15, positive for both *Mycoplasma hominis* and *Ureaplasma parvum*, microscopic cervicitis was not observed and microbiota was of supracytoplasmic bacilli (clue cells).

*Neisseria gonorrhoeae* was isolated in only one sample (sample 16) and with *Chlamydia trachomatis* (Table 1). The cytological findings were similar to that of the sample in which *Chlamydia trachomatis* was the sole pathogen detected: microscopic cervicitis with numerous polymorphonuclear leukocytes. Microbiota was normal (predominantly lactobacillary) (Table 1, Figures 3(c)–3(f)).

In sample with both *Chlamydia trachomatis* and *Ureaplasma parvum* (sample 17), microscopic cervicitis was not observed and microbiota was normal (predominantly lactobacillary).

### 3.3. Comparison between Liquid-Based and Conventional Preparations

Polymorphonuclear leukocytes were better distributed and less abundant in liquid-based preparation than in the conventional preparation. The microbiota was better evidenced in the preparations by the conventional method (Figures 3(c)–3(f)).

### 3.4. Comparison between Positive and Negative Samples in Multiplex PCR

In samples in which at least one pathogen was identified by multiplex PCR, microscopic cervicitis was observed in 88.2% (15/17) of the samples and in 100% (10/10) of the samples with normal microbiota (predominantly lactobacillary) (Table 1). In samples in which no pathogen was detected by multiplex PCR, microscopic cervicitis was observed in 60% (18/30) of the total samples and in 41.6% (5/12) of the samples in which the microbiota were normal (predominantly lactobacillary). Samples with at least one pathogen detected by multiplex PCR and with normal microbiota (predominantly lactobacillary) in cytology were compared with samples with no pathogen detected by PCR and normal microbiota in cytology to evaluate the presence of microscopic cervicitis. In samples with both microscopic cervicitis and normal microbiota, those with at least one pathogen identified by multiplex PCR were significantly more frequent than those with no pathogen, 66.6% versus 33.3% (Fisher's test *p* = 0.005), respectively.

### 3.5. Cycle Quantification (Cq) Values and Cytology

Positive cycle quantification (Cq) values ranged from 21.9 to 36.5 in samples in which at least one pathogen was detected. Microscopic cervicitis was observed even in samples in which pathogens were detected with Cq values > 33 (Table 1). *Trichomonas vaginalis*was observed on cytology only in samples with the lowest Cq values (21.9 and 24.2).

## 4. Discussion

All types of cytological specimens, namely, gynecological cytology, exfoliative nongynecological cytology, and fine needle aspirates can be used not only for cytological analysis but also for pathogen identification [8]. With cervical samples for liquid-based preparations, in addition to cytology, different molecular biology techniques can be applied to detect HPV and other sexually transmitted pathogens [9]. In the present study, cervical samples were collected for cytology and for detection of *Chlamydia trachomatis*, *Neisseria gonorrhoeae*, *Mycoplasma genitalium*, *Trichomonas vaginalis*, *Mycoplasma hominis*, *Ureaplasma urealyticum*, and *Ureaplasma parvum* by multiplex PCR.

*Mycoplasma genitalium* is considered, together with *Chlamydia trachomatis*, *Trichomonas vaginalis*, and *Neisseria gonorrhoeae*, a “true” sexually transmitted infection causing male urethritis and is associated with cervicitis and an increased risk of pelvic inflammatory disease, endometritis, and infertility in women [10]. *Mycoplasma hominis*, *Ureaplasma urealyticum*, and *U. parvum* are frequently found in the human urogenital tract in both healthy individuals and symptomatic patients [11, 12]. However, the relevance of the colonization/infections of *Mycoplasma hominis*, *Ureaplasma urealyticum*, and *Ureaplasma parvum*, which are among the opportunistic pathogens found in the urethral and vaginal flora, has yet to be determined [13, 14]. There are many questions about routine screening of asymptomatic men and women or routine testing of symptomatic individuals for *Mycoplasma hominis*, *Ureaplasma urealyticum*, and *Ureaplasma parvum* [14]. The extensive testing, detection, and subsequent antimicrobial treatment may result in the selection of antimicrobial resistance in these bacteria, in “true” STI agents, and in the general microbiota [14]. Studies to investigate unresolved issues regarding *M. hominis*, *U. parvum*, and/or *U. urealyticum* could be valuable [14].

Multiplex PCR was positive in 36.2% of the samples in the present study. *Ureaplasma parvum* was the most common pathogen 14.9%, followed by *Chlamydia trachomatis* 10.6%, *Trichomonas vaginalis* 10.6%, *Mycoplasma hominis* 8.5%, *Ureaplasma urealyticum* 4.2%, and *Neisseria gonorrhoeae* 2.1%. *Mycoplasma genitalium* was not detected in any of the samples. Multiple pathogens were observed in 12.8% of the samples. Previous studies have shown a great deal of variation in the prevalence of these pathogens in cervical samples, and this may be due to the different types of molecular tests employed and the population studied. In a previous study using multiplex PCR to detect the same pathogens in a large population of sexually active young women in Israel, 44.6% were positive for at least one pathogen. *Ureaplasma parvum* was identified in 28.2% of the samples followed by *Ureaplasma urealyticum* (15.7%), *Chlamydia trachomatis* (6.6%), *Mycoplasma hominis* (6.2%), *Mycoplasma genitalium* (1.9%), *Neisseria gonorrhoeae* (0.7%), and *Trichomonas vaginalis* (0.5%) [15].

Regarding cytology, the findings herein described were obtained from both conventional and liquid-based preparations. Nevertheless, since multiplex PCR detection was performed in liquid-based samples, only these were analyzed for type of microbiota and presence of microscopic cervicitis. Moreover, cell distribution is more homogeneous in liquid-based preparations compared to the conventional method, and regular distribution of cells facilitates their quantification. As expected, upon comparing the two methods in the present study, the number of polymorphonuclear leukocytes was higher, and the microbiota was more abundant when the conventional method was used.

The criterion for microscopic cervicitis (≥10 pmnl/epithelial cell) was established from samples with clinical diagnosis of mucopurulent cervical discharge. To the best of our knowledge, there is a lack of well-defined criteria for cervicitis on pap smears and, even more so, for pathogen prediction. In a previous study with liquid-based preparations, the authors concluded that using a threshold of ≥2 leukocytes per epithelial cell per high-powered field, the positive predictive values for *Mycoplasma genitalium*, *Chlamydia trachomatis*, *Neisseria gonorrhoeae*, and *Trichomonas vaginalis* were 100, 70, 67, and 20%, respectively [16]. The low threshold used in this previous study would explain the low positive predictive value of the method for *Trichomonas vaginalis* which usually causes intense inflammatory exudate.

Microscopic cervicitis (≥10 pmnl/epithelial cell) was present in 88.2% of the total samples with at least one pathogen detected and in 100% of the samples with both normal microbiota (predominantly lactobacillary) and at least one pathogen detected. Microscopic cervicitis was present in all samples in which *Ureaplasma parvum*, *Ureaplasma urealyticum*, *Chlamydia trachomatis*, and *Trichomonas vaginalis* were the sole pathogens detected. In the present study, *Mycoplasma hominis* and *Neisseria gonorrhoeae* were not found as the sole infecting pathogens, so it was not possible to assess the cytological findings related to each of these microorganisms individually. In two samples with multiple pathogens, sample 15 (*Ureaplasma parvum* and *Mycoplasma hominis*) and sample 17 (*Ureaplasma parvum* and *Chlamydia trachomatis*) microscopic cervicitis was not evidenced. This feature shows the importance of correlating PCR results to pap smear and clinical findings. The negative predictive value of microscopy tends to be high, since without polymorphonuclear exudate, there is probably no cervicitis [2].

There is disagreement between previous publications regarding the association between Ureaplasma load and the presence of cervicitis [5, 17]. The multiplex PCR used in the present study is qualitative and not quantitative. However, the cycle quantification (Cq) value could be used to estimate bacterial load; a low Cq value indicates a high load and vice versa [18]. Positive Cq values ranged from 21.9 to 36.5 in samples in which at least one pathogen was detected and microscopic cervicitis was observed even in samples in which pathogens were detected with Cq values > 33 (above the recommended cut-off Cq values for positive control).

Samples with both microscopic cervicitis and normal microbiota (predominantly lactobacillary) were compared for pathogen presence, and the results showed that microscopic cervicitis was significantly more frequent when at least one pathogen was identified by multiplex PCR. In samples in which no pathogen was detected by multiplex PCR and with normal microbiota (predominantly lactobacillary), the frequency of microscopic cervicitis was of 41.6% of the samples. In these samples, microscopic cervicitis may have been caused by a noninfectious inflammatory agent or by infectious agents not detected by the test. An unsatisfactory sensitivity of the test could also explain the presence of microscopic cervicitis in these cases. The test used here has the lowest sensitivity for *Mycoplasma genitalium*, and perhaps this is the reason for the lack of detection of this pathogen in any sample. In the diagnostic routine, by cytology the finding of intense neutrophilic exudate, without microbiota to justify this finding, is very frequent. Some samples are even categorized as unsatisfactory by pyocytes. The results of the present study suggest that at least in some of these cases, the cause may possibly be related to the presence of some pathogen, which could potentially be identified only by molecular tests or culture. According to the Bethesda system, it is optional to report organisms or other nonneoplastic findings in cervical cytology. However, in such cases, the intensity of inflammation should be mentioned so that it could be correlated with clinical data and PCR results.

With respect to microbiota, in samples with pathogens identified by PCR, the normal microbiota (predominantly lactobacillary) were the most frequent (58.8%, 10/17) followed by coccobacilli and supracytoplasmic bacilli. It is noteworthy that samples with potential inflammatory agents such as *Candida sp* and actinomyces and with cytopathic effects consistent with herpes and cytomegalovirus were excluded from this study, as these pathogens could be the cause of inflammatory cytological changes. The presence of these microorganisms would not allow the association analysis between microscopic cervicitis and the presence of pathogens identified by multiplex PCR. Similarly, only samples with normal microbiota were used in the analysis of the association between microscopic cervicitis and the presence of at least one pathogen in the multiplex PCR, because there are several studies showing that the coccobacillary microbiota, mainly aerobic bacteria, can be associated with the presence of inflammation [19, 20].

*Trichomonas vaginalis* was identified only by PCR in 3 out of 5 samples. This disagreement between cytology and PCR for identification of this pathogen was expected since molecular techniques are more sensitive than microscopy for detection of *Trichomonas* vaginalis [21]. The presence of *Trichomonas vaginalis* on cytology was only identified in samples with the lowest Cq values (21.9 and 24.2). This would be expected since low Cq values are associated with high pathogen load. In fact, if the highest Cq from a sample where *Trichomonas vaginalis* could still be detected by microscopy was taken as baseline (24.2), comparisons with other samples could be drawn. For instance, samples where Trichomonas microscopical identification was not possible showed Cq values of 31.27, 35.1, and 36.53 corresponding to a pathogen load 132x, 2320x, and 5077x, respectively, lower than the sample where microscopy identification was feasible. Taken together, these results confirm the diagnostic power of the PCR technique.

The microbiota was normal (predominantly lactobacillary) in the sample with *Neisseria gonorrhoeae*, and diplococci were not evidenced. Identification of *Ureaplasma* ssp, *Mycoplasma* ssp, and *Chlamydia trachomatis* would not be expected in pap smear because they are not visible through light microscopy. Ureaplasmas are coccobacillary-shaped bacteria with diameters between 0.2 and 0.3 *μ*m and the lack of a rigid cell wall impairs its visualization. [22] The elementary body, which is the extracellular form of *Chlamydia trachomatis*, has a diameter of only 0.3 *μ*m [23].

In addition to features related to inflammation and microbiota, in two samples in which *Trichomonas vaginalis* was detected, HSIL was also identified. The association of pathogens of sexually transmitted diseases with HPV infection and cytological abnormalities has been described in the literature [24, 25]. Although pap smear is used for cancer and its precursor lesion screening, it may be considered predictive for pathogens since screening patients through more accessible diagnostic methods, such as pap smears, may be the only option in less developed countries.

## 5. Conclusion

Cervical pap smear findings are nonspecific and characterized by intense inflammation and normal microbiota (predominantly lactobacillary) in most samples in which at least one pathogen was identified by multiplex PCR. Failure to identify an inflammatory agent in cervical pap smear with intense neutrophil exudate may suggest the presence of *Ureaplasma parvum*, *Ureaplasma urealyticum*, *Chlamydia trachomatis*, or *Trichomonas vaginalis*. A remark on the intensity of inflammation should be made in the reports of cervical pap smears so that this cytological finding can be correlated with clinical and PCR results.

## Figures and Tables

**Figure 1:** Liquid-based preparation of sample from patient with mucopurulent discharge (control sample). (a) Homogeneous cell distribution of epithelial squamous cell and polymorphonuclear leukocytes (pmnl). Numerous pmnl, isolated (b) and in aggregates (“polyballs”) (c). (d) Normal microbiota (lactobacilli) (orange arrow). Papanicolaou: (a) 100x, (b, c) 400x, and (d) 1000x.

**Figure 2:** Cervical cytology of samples in which *Ureaplasma parvum* (a, b), *Ureaplasma urealyticum* (c, d), *Chlamydia trachomatis* (e, f), and *Trichomonas vaginalis* (g, h) were the sole detected pathogen by multiplex PCR. Numerous polymorphonuclear leukocytes isolated and in aggregates (“polyballs”) (a–h). Normal microbiota (lactobacilli) in (b, d, f) (bottom right corner). (h) Pear-shaped organism with eccentrically located nucleus and eosinophilic cytoplasmic granules, consistent with *Trichomonas vaginalis* (orange arrow in upper right corner) and HSIL (yellow arrow). Papanicolaou: (a) 200x; (c, g) 100x; (b, d, f, h) 400x; (e) 40x; (bottom right corner) 1000x. (a–d, g, h) Liquid-based; (e, f) conventional cytology.

**Figure 3:** Cervical cytology of samples with multiple pathogens detected by multiplex PCR: (a) *Mycoplasma hominis* and *Trichomonas vaginalis* (sample 14); (b) *Mycoplasma hominis*, *Trichomonas vaginalis*, and *Ureaplasma parvum* (sample 12); (c–f) *Chlamydia trachomatis* and *Neisseria gonorrhoeae* (sample 16). Numerous polymorphonuclear leukocytes, isolated and in aggregates (“polyballs”) in (a–f). Pear-shaped organisms with eccentrically located nucleus and eosinophilic cytoplasmic granules, consistent with *Trichomonas vaginalis* (green arrow) and HSIL (red arrow) in (a). Coccobacilli (blue arrow) and spermatozoid (yellow arrow) in (b). (c–f) Numerous polymorphonuclear leukocytes in mucus were better distributed and less abundant in liquid-based (e, f) than in conventional preparation (c, d). Normal microbiota (lactobacilli) is less abundant in liquid-based preparation (e, f) than in conventional preparation (c, d). (f) Lactobacilli (upper right corner, orange arrow). Papanicolaou: (a, e) 200x; (b) 1000x; (c) 100x; (c, f) 400x; (upper right corner) 1000x. (a–d) Conventional cytology; (e, f) liquid-based cytology.

**Table 1:** Cervical samples with pathogens identified by multiplex PCR with respective Cq values and cytological findings (microbiota and presence of microscopic cervicitis).

Sample number	Uparv	Uurea	CT	Tvag	Mhom	MG	GC	Microbiota	Microscopic cervicitis
1	35.2							Lactobacilli	x
2	31.1							Supracytoplasmic bacilli	x
3	34.3							Lactobacilli	x
4	31.3							Lactobacilli	x
5		30.8						Supracytoplasmic bacilli	x
6		27.9						Lactobacilli	x
7			31.9					Coccobacilli	x
8			24.6					Lactobacilli	x
9			24.6					Lactobacilli	x
10				24.2				Coccobacilli	x
11				36.5				Lactobacilli	x
12	33.8			35.1	33.6			Coccobacilli	x
13				31.2	31.3			Lactobacilli	x
14				21.9	22.9			Coccobacilli	x
15	32.6				34.7			Supracytoplasmic bacilli	
16			34.1				35.4	Lactobacilli	x
17	35.8		28.1					Lactobacilli	

CT: *Chlamydia trachomatis*; GC: *Neisseria gonorrhoeae*; MG: *Mycoplasma genitalium*; Tvag: *Trichomonas vaginalis*; Mhom: *Mycoplasma hominis*; Uurea: *Ureaplasma urealyticum*; Uparv: *Ureaplasma parvum*.

## Data Availability

All materials and data are fully described within the manuscript.
